This article has been retracted.

# The Commitment of Nineveh Governorate Residents to the Precautionary Measures against Global 2019 Pandemic and Dermatological Affection of Precautions

**DOI:** 10.1155/2021/1526931

**Published:** 2021-12-13

**Authors:** Baraa A. Al-Rahawe, Abdulsattar Abdullah Hamad, Mohanad H. Al-Zuhairy, Hameed Hasan Khalaf, Solomon Abebaw

**Affiliations:** ^1^Specialty of Biology, Gifted School of Nineveh, Gifted Guardianship Committee, Directorate of Education, Mosul, Iraq; ^2^College of Sciences Tikrit University, Iraq; ^3^Tikrit University, Iraq; ^4^Department of Statistics, Mizan-Tepi University, Ethiopia

## Abstract

The world has changed dramatically since the novel pandemic pours in all aspects of life, including economic, health, and social life. The first case was initially observed in the Wuhan province of China; fast spread occurs around the world. Until now, there is no proven effective treatment for it. The study's objectives are to assess residents of Nineveh governorate's commitment to the COVID-19 pandemic precautionary measures recommended by the WHO and Iraqi national authorities; the protective measures are used to prevent its spread and restrict the viral infectivity. Several cutaneous changes were observed in some persons as a result of prolonged contact with personal protective equipment and excessive use of personal hygiene measures.

## 1. Introduction

The COVID-19 first discovered case was on December 2019, Wuhan, China, as a cluster of nonclassical pneumonia with symptomatic and asymptomatic infections reported [1]. The first case reported in Iraq was on the 24 February 2020 in Najaf before 27 days of the first case reported in Nineveh [2]. On 9 January 2020, the Chinese government reported that the cause of the outbreak was a novel coronavirus, recently named SARS-CoV-2, as it is 80% identical to the previous SARS-CoV [1]. The WHO declared COVID-19 as the sixth public health emergency of international concern on 30 January 2020 due to its high respiratory transmission efficiency from person to person leading to rapid spread of the epidemic [3]. The causative is a zoonotic virus, a new strain of positively sensed single-stranded RNA viruses enveloped by large pleomorphic spherical particles with bulbous surface projections (spike glycoprotein) [1]. Until the time of writing this research, 8 March 2021, the COVID-19 pandemic has led to more than 117 million cases and 2 million deaths worldwide [3], and at the same time, in Iraq, there are 726,548 confirmed cases and 13,572 mortalities recorded [2].

We are learning more about how COVID-19 affects people every day. A study suggests that the novel coronavirus-2 could remain in the air for up to 3 hours post podsolization [4]. Another study, done in Wuhan hospitals, tested the air during the COVID-19 outbreak; results raise the suspicion of aerosol transmission of the virus [5]. Human-to-human transmission of SARS-CoV-2 occurs in a similar way to flu transmission through direct contact with respiratory droplets (coughing and sneezing) especially if the healthy person is close standing within one meter from the COVID-19 patient. Individuals can also be infected by touching surfaces contaminated with the virus and touching their faces (eyes, noses, or mouths) [6–8]. COVID-19 infects the upper and lower part of respiratory tract mucosa, while conjunctiva with the optic canal has the lowest risk of transmission. The incubation period has been estimated to be 14 days on average, while most of the cases show symptoms in 4 to 5 days from exposure and can be infected with mild or even no symptoms [9, 10].

Fever was the most common symptom, followed by sore throat, dry cough, aches, headache, and general weakness with breathing problems ranging from flu-like illness symptoms to pneumonia, severe acute respiratory distress syndrome, and sepsis septic shock leading to lung failure in more serious cases that require treatment with oxygen and a ventilator or even lung transplants reported in few COVID-19 patients [11]. Other symptoms that are less common include loss of taste or smell, diarrhea, skin rash, nasal congestion, and redness of the eyes. About 82% of people who have COVID-19 get mild to moderate symptoms or even asymptomatic, while about 14% of COVID-19 cases are severe and fatality rate of 3.4% in advance age, immune-compromised state, and presence of chronic medical conditions those considered as risk factors for serious illness as estimated by the WHO up to March 2020 [12, 13]. Another possible complication of a severe case of COVID-19 is that occurs when an infection reaches and spreads through the bloodstream causing tissue damage everywhere it goes, leaving the body more vulnerable to infection with another bacterium or virus [14]. There is evidence that 20-30% of critically ill patients can develop clots in the lungs, heart, brain, and lower extremities, some of which are life-threatening. So even if death does not occur in COVID-19, some patients survive with permanent lung damage [15, 16]. Still, there are ongoing studies to find whether these effects are permanent or might heal over time [17–19].

Based on the 2003 Severe Acute Respiratory Syndrome (SARS) and Middle East Respiratory Syndrome (MERS) epidemic experiences, elimination of the source of infection, early diagnosis, reporting, isolation, obliging the population to house quarantine, increase public awareness about the viruses, handwashing, and wearing protective masks play an important role in the controlling of the outbreaks [20]. Effective personal protective measures established by the WHO are as follows: avoiding close, crowded places and close contact to others for less than 2-meter safe distance with promoting personal protection to masks to reduce the risk of infection transmission when they cough, sneeze, or speak. The recommended mask by the WHO for the public to use is the nonwoven composed of oriented or random fabric mask, particularly in crowded and poorly ventilated places. Masks are made of the polymer extruded and stretched to form continuous filaments, laid into a web bonded by itself, while respirator masks (such as FFP2, FFP3, N95, and N99) made of 3 layers should be used where procedures generating aerosols are performed for maximum 8 hours of wearing and using wipes to cough or sneeze in them. Wearing gloves were not included as protective equipment by the WHO [21] unless by the Iraqi national health authorities [2]. Surgical gloves are made of different polymers including latex, nitrile rubber, polyvinyl chloride, and neoprene, coming unpowered or powdered with modified corn starch or calcium carbonate to lubricate the gloves, making them easier to put on [40]. Corn starch replaced tissue-irritating lycopodium powder and talc, but it also can impede healing if it gets into tissues.

In many places throughout the world, injuries constitute a leading cause of preventable mortality. More than 6 million people died as a consequence of accidental injuries in the year 2000, including 3.8 million accidental and 2.2 million deliberate injuries (1). In many nations, the spectrum of mortality and illnesses has shifted in recent decades (2, 3), and injury-related fatalities have become a major issue. The majority of injuries are avoidable, and in many affluent nations, injury prevention has been made a national priority, and accident-related mortality has been gradually declining for many years. A priority is to acquire additional data on damage and ill-health caused by unintentional injuries. Injuries account for around 12% of the world's illness burden (5). Injuries, regardless of their source or aim, have a significant impact on the health care system that offers care and assistance to victims (6). The impact of trauma is poorly recognized in many developing nations, notably in Asia, because of a lack of health statistics recording.

However, cleaning hands regularly and thoroughly with the ethanol or isopropyl alcohol hand rub with 70% concentration was recommended by the WHO and the Iraqi health ministry or washing them with soap and water to eliminate germs sticking to them including viruses. Ensure regular physical activity and incarnate vitamins and minerals supplement through healthy food or pills to enhance the immune system in fighting infections, keeping up to date on the latest information of protective measures and vaccination from reliable sources of disease [16]. There is an establishing vaccination; however, they still need further trials with more time to be proved as a safe, effective treatment to control the COVID-19 pandemic and to deal with its side effects [22–24]. For that, the control measures and healthy lifestyle with an efficient immune system are the only safe and proven ways to reduce SARS-CoV-2 spreading.

## 2. The Aims of the Study

The study's objectives are to assess residents of Nineveh governorate's commitment to the COVID-19 pandemic precautionary measures recommended by the WHO and Iraqi national authorities, as there has been no previous research conducted within Iraq or Nineveh governorate to provide information about the population's knowledge and practice of protective measures, which would help to bridge the gap between perception and practice.

To determine if there is any dermatological ailment, use protective equipment (e.g., masks, gloves, and alcohol sanitizer) and the chemical ingredients are comprised.

If a dermatological condition has appeared, identify the locations, indicators, and causative agents.

## 3. Materials and Methods

### 3.1. Conceptual Framework and Study Design

We conducted a prospective cross-sectional survey between September 1 and November 31, 2020, at Nineveh governorate, Iraq. In an epidemiological study, the goal of this researches is to figure out the epidemiology of injury-related mortality in the Nineveh governorate. Methodology: in order to assess the epidemiology of mortality from accidents in the Nineveh governorate, a retrospective analysis was used. There are 5707 men, 4180 females, and 1527 females in the sample. The research was conducted over a five-year period, beginning in the year 2000 and ending in the year 2005 (2008 to 2012). The sample ranged in age from 1 to 65 years old. Data was gathered from the Forensic Medicine Center, the Nineveh Governorate's Primary Health Care Sector, and the Nineveh Health Department. it is well known that it is so difficult to involve all the population in the community; therefore, we conduct our study depending on randomized sampling through using 27 questions, Arabic written paper, and online google form questionnaires to describe the studied community within the accepted statistical values. We have designed the survey's questions into three aspects according to the goals we want to reach in our research and as multiple-choice questions as being easier to answer, hence having proper and useful information from the sample. At the top of the questionnaire, there was an introductory part that encompassed the purpose and objectives of the study and consent information to ensure voluntary participation in the study as well as participant anonymity and confidentiality. The first section of the form was about the general health and socio comic's information for the inclusivity purpose of sample. The second section was including 16 questions of precautionary measures against COVID-19 recommended by the WHO and the Nineveh governorate authorities pandemic graded as always 100% to 80% of time, often 79% to 20% of time, or rarely 19% or less of time committing to them to evaluate the degree of the obedience of Nineveh residents to them, while adding more options will lead to confusion and misunderstanding to the fine difference between them. The third section was subedited to know if there is any sign of dermatological affection related to using precautionary measures that appeared; it is the type and the causative. The questions of this section are shown in Table 1.

What is the type of hand disinfectant you are using? How many times are you using it weekly? Has any sign of dermatological affection appeared on you because of using the precautionary equipment? What is/are the site/s of dermatological affection you have experienced because of using the precautionary equipment? And what is/are the sign/s of the dermatological affection you have experienced?

### 3.2. Sample Collection

Initially, only citizens of the Nineveh governorate participated, with a total of 1218 participants. The paper questionnaires were distributed and published in medical clinics, government companies, and online through various social media platforms (Facebook and Telegram), and participants were only allowed to answer them 1once to ensure wide distribution to the target population, good coverage of respondents from various socioeconomic backgrounds, and the accuracy of the results we have reached. The questionnaire and replies, once gathered and processed, were freely accessible to participants. They were anonymous surveys, and recording or dissemination did not generate identifiable information. The sample of the research has included both gender, all age groups, different occupations, and from different areas within the Nineveh governorate. As shown in Table 1, the median age was between 31 and 40 years and 511 (56.3%) were male. Of these patients, 300 (33.1%) were students, and 599 (66.0%) were from the city center (Mosul city).  Table 2 also demonstrates the distribution of the participants regarding the history of medical illness, the highest percentage being 72% that is the healthy persons; other chronic diseases were present in different percentages.

### 3.3. Statistical Method and Data Analysis

311 of the involved participants were excluded from the total 1218 because of inaccuracy in their answers and lack of complete information. So we had a total of 907 sample participants included in the research. The information obtained from questionnaires was analyzed into a statistical form using SPSS (Statistical Package for the Social Science) version 25.0 (IBM Corp, Armonk, NY) after converting this information to the codec required by the program according to each question criteria, while most of the questions were three codec answers (always, often, and rarely). In addition, we have used the Excel sheet.

## 4. Results

From the analysis of data given by our sample about the first section of the questionnaire which was direct to the commitment of Nineveh governorate residents to the precautionary measures against COVID-19 pandemic, in Table 3, we have had the following result.

From all questions we have asked the participant previously, we came to the final median of Nineveh governorate resident commitment to the precautionary measures against COVID-19 pandemic that we have concerted on in the first section of the research and the result is as in Table 4.

As Table 4 demonstrates, 42% of Nineveh residents were always committing to the precautionary measures, and 40% were often committing them, while 18% were not committing them as they have to.

When it comes to the second component of the study and the questionnaire, which was about the dermatological effects of utilizing protective gear on the Nineveh residents, governorate residents, we have had the results shown in Table 5.

From the 907 participants we had, about 80% of them have not shown any dermatological allergy signs while the remaining 21% have expired dermatological affection of using these precautionary measures which are about 186 participants (Table 5).

About the place of affection, 77% of the affected 186 participants have experienced the manifestation in their hands (palm and back), 13% in their faces (cheeks and periorbital skin as it is the thinnest cutaneous found in the face), and 6% in their noses (nose bridge), and the lowest percentage (4%) of the affected participants has experienced the manifestation in their per orbital skin (Tables 6 and 7).

In Table 2, 41 participants of the 186 affected participants (33%) have shown dermatological affection in their faces (cheek, nose, and periorbital), and 66% of them were wearing masks always, and 32% were often wearing masks, while only 2% were doing so rarely. Wearing a mask can cause pressure urticarial, contact dermatitis, itching, indentations, and acneiform eruption.

About third of the cutaneous manifestation that appeared on their skin was itching, 32% was redness as it is the first sign of allergen, 26% was excoriation of the skin, and the remaining was edema or other signs, i.e., scaling, itching, irritation, and skin maceration (Table 8).

## 5. Discussion

To our knowledge, this is one of the few community-based studies dealing with residents' commitment to personal safety precautions and the dermatology effects of personal protective equipment (PPE) utilized in the Nineveh governorate. The results of this study reveal that, on average, people follow the WHO's and other relevant national and local agencies' directions. While earlier studies have concentrated on the knowledge, awareness, and practice (KAP) of concerned populations, we have endeavored to include practically all preventative measures against coronavirus 2019. More knowledge of the risk of COVID-19 infection is noticed in the city center, a densely populated location compared to rural areas, and a high socioeconomic standard might explain this obedience.

The middle-aged participants have shown more commitment to the precautionary measures that may be related to more knowledge as most of them were teachers and highly educated employers; in addition, this age group is usually complaining from chronic diseases which are considered as a risk factor for morbidity and mortality with COVID-19 [25]. Analysis of the data reveals a variable degree of adherence to each item of the protective measures involved in the survey's questions, with the higher result being with the use of facial masks and avoiding crowded places as they are the main defense measures against aerosol SARS-CoV-2; also with respond to house quarantine that has been imposed by Nineveh health authorities, this corresponds to the result obtained by Kwok et al. in Bangladesh [8] due to the obligatory law by governments and censorship in public places. Information from the data obtained shows that female participants are more obeying the protective instruction than males corresponding to a study carried out in Karachi, Pakistan [26]. Wearing gloves, adding food supplements to their diet, avoiding mass transport, and cloth sterilizing were the lowest committed precautions, respectively; higher cost of the personal transportation cars (taxis) and the need for medical prescription for vitamins and minerals could explain these findings. Relative studies done in Saudi Arabia, Bangladesh, China, and Malaysia have shown similar findings about community knowledge and consciousness to the essential hand hygiene and wearing gloves [27–30]. However, only 10% of people in Nineveh keep aware of up-to-date information from reliable sources about COVID-19. Eating house made foods with washing fruits and vegetables thoroughly has shown mild obedience results. Washing hands with soap and water or using hand detergents demonstrated a noticeable commitment (41%). This precautionary measure was also highly adherence by the Saudi (97%) and Chinese communities [31, 32]. These in line findings with previous studies may be explained as that these protective behaviors are the second main way to break the transmission chain of most infectious diseases and control infection rates, while the commitment of Nineveh residents to washing hands with soap and water in 5 steps for more than 20 seconds which is the effective way recommended by the WHO was 31%, being higher than what the Saudi research finds (only 1 in 7 is washing hands using the protocol recommended by the WHO) [27]. This difference could be explained by the natural concept of our community regarding the proper way of washing hands rather than depending on expensive disinfectant as a method for viral elimination. More than half (51%) of Nineveh residence have been using disposable wipes while sneezing or coughing, 35% of them have been getting rid of precautionary equipment in a proper way, and 27% are frequently doing sports activities.

On the other hand, the majority of participants have not shown any cutaneous manifestations following using precautionary equipment (i.e., gloves, masks, and disinfectants) for those who develop cutaneous manifestations; female participants are affected more than males; this could be due to the excessive use of the precautionary measures by the female group. Regarding the dermatological manifestations, there is mild skin affection among those who use detergents with the highest incidence (77%) being in the skin of the hands and less frequent in the face (nose and periorbital skin). Other researches are done by Masood et al., and Darlenski and Tsankov have shown that the nasal bridge and facial irritation is the more widespread than hand irritation in health care workers (HCWs); this discrepancy is explained by the fact that the above researches were done among the HCWs, those using facial respirator masks and goggles for a long period of time [33, 34]. Hand lesions are caused mainly by the frequent and overusing of high concentration (70% and more) alcohol sanitizer as it was the commonest disinfectant against SARS-CoV-2 in comparison to less frequent hand protective measures like wearing surgical gloves shown in only 15% percent of hand lesion affected participants due to excessive use of it instead of washing hands with water as about half of hand affected persons were using the alcohol sanitizer more than 35 times weekly as being less expensive, highly available, and easily handled everywhere; in addition, it is recommended by the WHO as a part of precautionary equipment for COVID-19. Based on these results, we can say that the appearance of these lesions is directly proportionate to the duration of contacting skin to alcohol, the frequency of its use as there are the main determinant factors in the development of the cutaneous manifestations, which support the idea mentioned above. Alcohol sanitizer and the other used disinfectants are chemical substances that affect the hydrolipid barrier causing dryness and irritation; the allergenic components of the gloves, presence of irritant powder, and the loss of humidity due to prolong use can give the reason behind this finding. Cutaneous lesions are commonly manifested as itching and redness as they are the first sign of allergic response. About 65% of the dermatological lesion affected participants have been shown in the persons who wear masks always that create pressure and abrasion and maintain a moist environment which leads to skin changes mainly at cheek level, periorbital, nasal bridge, and other prominent facial areas. Using alternative protective equipment characterized by their low contact to the skin such as face shields can reduce that irritation shown. Other previous study done by Masood et al. suggests applying a good barrier cream (e.g., Vaseline and petroleum jelly) before and after wearing PPE as skin scaling and dryness are very common because of humid and close environments due to water in exhaled air that can impair the skin barrier function causing pressure urticarial, contact dermatitis, itching, indentations, acne, folliculitis, and exacerbate seborrheic dermatitis [33].

## 6. Conclusions and Recommendations

1. We can reduce the skin affection through limitation of using of alcohol or use low concentrated alcohol with same efficacy if possible
2. This study was conducted during the peak of pandemic that explains the high commitment of the participants with the protective measures; we expect that the people in Mosul city will become less interested with protective measures as they thought that the infection regress, or there is no benefit from using these measures, or become boring from overuse, the availability and accessibility of the COVID-19 vaccination in addition to the financial aspect and other causes
3. More studies are needed to find the causes behind that refusal or nonobeying the health instructions among some people in our locality and to manage those causes accordingly
4. Further prolonged studies are also needed to determine the long-term squally of using protective measures (gloves, disinfectant, and facial mask)
5. Frequent change of facial masks and gloves with the use of disposable on
6. Manufactured protective tools like masks and gloves with a less allergen substance
7. Using all the available governorate resources to encourage social distance concept application in the places suspected to be overcrowded
8. Encourage people to use skin protective tools to wash their skin more frequently with water as it is the basic and most effective preventive measure against infection; it also eliminates the allergic effect of the alcohol and latex of the gloves which result from prolonged exposure to these allergens
9. We expect that there are gaps between perception and practice and would allow decision-makers and public health authorities to evaluate the awareness of these preventative measures in order to address any deficiencies by suitable targeted means and campaigns
10. Based on the previous results, and for reducing the economic burden, also preventing the overcontact of the allergen, i.e., alcohol, we suggest to avoid the excessive use of alcohol as it is the main causative factor of the detected cutaneous lesions, with or a shelled washing hands
11. Need for dermatologists and health instructions to increase the public awareness and knowledge about the dermatological affection of protective measure they are using every day and how to reduce this affection and adapt them in a proper way

## Figures and Tables

**Table 1:** General sociodemographic information of research participant.

General information	Choice	Number of participants (% of involved participants)
Gender	Male	511 (56.3%)
	Female	396 (43.7%)
Age distribution	10 to 20 years	84 (9.3%)
	21 to 30 years	173 (19.1%)
	31 to 40 years	182 (20.1%)
	41 to 50 years	194 (21.1%)
	51 to 60 years	172 (19.0%)
	Older than 60 years	102 (11.2%)
Residence	City center	599 (66.0%)
	Subdistrict	181 (20.0%)
	District	172 (14.0%
Occupation	Student	300 (33.1%)
	Lecturer	23 (2.5%)
	Housewife	164 (18.1%)
	Doctor	35 (3.9%)
	Free business	152 (16.8%)
	Retired	20 (2.2%)
	Teacher	28 (19.3%)
	Officer	185 (20.4%)
Chronic disease	None	705 (77.7%)
	Diabetes mellitus	22 (2.3%)
	Hyperlipidemia	16 (1.8%)
	Thyroid disorder	11 (1.2%)
	Atherosclerosis	12 (1.3%)
	Sinusitis	9 (1.0%)
	Allergy	19 (2.1%)
	Bronchial asthma	32 (3.5%)
	Heart failure	8 (9.0%)
	Hypertension	63 (6.9%)
	Renal impairment	11 (1.2%)

**Table 2:** The relationship between wearing a mask and face dermatological manifestation shown in the 43 participants.

	Choice	Number of face dermatological manifestation participants responded (of face affected participants) (%)
Relationship between wearing mask and face dermatological manifestation shown in the participants	Always	27 (65.8%)
	Often	13 (31.7%)
	Rarely	1 (2.5%)

**Table 3:** Responses of Nineveh governorate residence to each precautionary measure recommended by the WHO and imposed by the national authorities.

Precautionary measure	Choice	Number of participants responded (%)
Do you commit to wearing a mask when you go out or in crowded unventilated spaces?	Always	604 (67.0%)
	Often	256 (28.0%)
	Rarely	47 (5.0%)
Do you commit to keeping 2-meter safe distance from others?	Always	306 (33.7%)
	Often	525 (57.9%)
	Rarely	76 (8.4%)
Do you commit to wearing gloves when you are outside your house?	Always	604 (66%)
	Often	256 (28.2%)
	Rarely	47 (5.2%)
Do you commit to avoiding crowded, closed, and unventilated places?	Always	612 (67.5%)
	Often	249 (27.5%)
	Rarely	46 (5.1%)
Do you commit to using hand detergents or washing your hands with soap after touching things outside your house?	Always	369 (40.7%)
	Often	505 (55.7%)
	Rarely	33 (3.6%)
Do you commit to washing your hands for at least 20 s and in the 5 steps way recommended by the WHO?	Always	279 (30.8%)
	Often	430 (47.4%)
	Rarely	198 (21.8%)
Do you commit to house quarantine being imposed by health and directorial governorate authorities?	Always	601 (66.3%)
	Often	260 (28.7%)
	Rarely	46 (5.1%)
Do you commit to sterilizing or washing your clothes when you return to your house?	Always	60 (6.6%)
	Often	310 (34.2%)
	Rarely	537 (59.2%)
Do you eat takeout foods from restaurants and cafes?	Always	51 (5.6%)
	Often	268 (29.5%)
	Rarely	588 (64.8%)
Do you use the mass transportations when you are transporting from one place to another?	Always	108 (11.9%)
	Often	276 (30.4%)
	Rarely	523 (57.7%)
Do you commit to washing fruits and vegetables before eating them?	Always	594 (65.5%)
	Often	289 (31.9%)
	Rarely	24 (2.6%)
Do you commit to doing sports activities to enhance your immune system and health?	Always	244 (26.9%)
	Often	388 (42.8%)
	Rarely	275 (30.3%)
Do you commit to doing sports activities to enhance your immune system and health?	Always	244 (26.9%)
	Often	388 (42.8%)
	Rarely	275 (30.3%)
Do you use food supplements of vitamins and minerals that improve your immunity?	Always	148 (16.3%)
	Often	418 (46.1%)
	Rarely	341 (37.6%)
Do you use disposable wipes when you are sneezing or coughing?	Always	454 (50.7%)
	Often	383 (42.8%)
	Rarely	58 (6.5%)
Do you commit to getting rid of precautionary equipment in the right way recommended by the WHO?	Always	317 (35.0%)
	Often	480 (52.9%)
	Rarely	110 (12.1%)
Do you commit to being aware of up-to-date information about COVID-19 and precautionary measures from the WHO and national health authorities?	Always	317 (35.0%)
	Often	480 (52.9%)
	Rarely	110 (12.1%)

**Table 4:** Evaluation of Nineveh governorate residence commitment to the precautionary measures.

	Degree of obedience	Number of participants responded (%)
The overall commitment of Nineveh governorate residents to the precautionary measures	Always	377 (41.6%)
	Often	368 (40.5%)
	Rarely	162 (17.9%)

**Table 5:** The participants have shown dermatological affection of the total involved participants.

Question	Choice	Number of participants responded (%)
Have you experienced any dermatological manifestation?	Yes	186 (20.5%)
	No	721 (79.5%)

**Table 6:** The sites of dermatological affection 186 of our total participants have experienced.

Question	Choice	Number of participants affected (%)
What is/are the site/s of dermatological affection that have shown in your skin?	Hands	143 (76.9%)
	Periorbital	7 (3.7%)
	Face	25 (13.5%)
	Nose	11 (5.9%)

**Table 7:** The relationships between hand dermatological manifestation and possible cause for it in the 143 participants.

	Choice	Number of hand dermatological manifestation participants responded (of hand affected participants) (%)
The relationship between the type of hand disinfectant and the hand dermatological affection shown	70% alcoholic sanitizer	90 (63.2%)
	DETTOL	35 (24.3%)
	Hand hygiene	18 (12.5%)
The relationship between the frequency of using hand disinfectant and the hand dermatological affection shown	1 to 7	1 (0.7%)
	8 to 14	3 (2.0%)
	15 to 21	7 (4.9%)
	22 to 28	23 (15.4%)
	29 to 35	39 (27.3%)
	More than 35	71 (49.7%)
The relationship between wearing gloves and the hand dermatological affection	Always	22 (15.6%)
	Often	56 (39.1%)
	Rarely	65 (45.3%)

**Table 8:** The sign/s of the dermatological manifestation shown in the 907 participants.

	Choice	Number of hand dermatological manifestation participants responded (of hand affected participants) (%)
The sign/s of dermatological affection shown in the participants	Excoriation of skin	39 (25.9%)
	Odema	13 (7.7%)
	Redness	48 (32.2%)
	Itching	49 (32.8%)
	Others	4 (1.4%)

## Data Availability

The data underlying the results presented in the study are available within the manuscript.
